The article "Carbapenem Resistance and Acinetobacter baumannii in Senegal: The Paradigm of a Common Phenomenon in Natural Reservoirs" was retracted in 2025. Reasons: lack of ethics approval or compliance; missing or withdrawn patient consent; concerns about the data; concerns about the welfare of human subjects.

# Carbapenem Resistance and *Acinetobacter baumannii* in Senegal: The Paradigm of a Common Phenomenon in Natural Reservoirs

**DOI:** 10.1371/journal.pone.0039495

**Published:** 2012-06-20

**Authors:** Marie Kempf, Jean-Marc Rolain, Georges Diatta, Saïd Azza, Bissoum Samb, Oleg Mediannikov, Amy Gassama Sow, Seydina M. Diene, Florence Fenollar, Didier Raoult

**Affiliations:** 1 Unité de recherche sur les maladies infectieuses et tropicales émergentes (URMITE), UMR CNRS-6236, Aix Marseille Université, Marseille, France; 2 Institut de Recherche pour le Développement, URMITE, Dakar, Sénégal; 3 Unité de Bactériologie Expérimentale Institut Pasteur, Dakar, Sénégal; Charité, Campus Benjamin Franklin, Germany

## Abstract

Incidence of carbapenem-resistant *Acinetobacter baumannii* is rising in several parts of the world. In Africa, data concerning this species and its resistance to carbapenems are limited. The objective of the present study was to identify the presence of *A. baumannii* carbapenem-resistant encoding genes in natural reservoirs in Senegal, where antibiotic pressure is believed to be low. From October 2010 to January 2011, 354 human head lice, 717 human fecal samples and 118 animal fecal samples were screened for the presence of *A. baumannii* by real time PCR targeting *bla*_OXA51-like_ gene. For all samples positive for *A. baumannii*, the carbapenemase-hydrolysing oxacillinases bla_OXA23-like_ and bla_OXA24-like_ were searched for and sequenced, and the isolates harbouring an oxacillinase were genotyped using PCR amplification and sequencing of *rec*A gene. The presence of *A. baumannii* was detected in 4.0% of the head lice, in 5.4% of the human stool samples and in 5.1% of the animal stool samples tested. No *bla*_OXA24_ gene was detected but six fecal samples and three lice were positive for *bla*_OXA23-like_ gene. The *bla*_OXA23-like_ gene isolated in lice was likely a new oxacillinase sequence. Finally, the *A. baumannii* detected in stools were all of *rec*A genotype 3 and those detected in lice, of *rec*A genotype 4. This study shows for the first time a reservoir of *bla*_OXA23-like_-positive gene in human head lice and stool samples in Senegal.

## Introduction

*Acinetobacter baumannii* is a Gram-negative coccobacillus that has emerged over the last few decades as a cause of both healthcare-associated and community-acquired infections [1], [2]. This bacterium is an important nosocomial pathogen of critically ill patients that can cause a wide range of infections, including ventilator-associated pneumonia, bloodstream infections, wound infections and nosocomial meningitis [1], [3], [4]. While *A. baumannii* is isolated from patients and hospital environment sources during outbreaks, the reservoir outside hospitals is not well delineated. This species can be isolated from human skin (between 0.5% and 3% according to the study), animal feces, water, soil or vegetables [5]–[8], but taken together, current data indicate that occurrence of *A. baumannii* in the environment is not well characterized [9]. The bacterium has also been isolated from human head and body lice as previously described [10].

Acquired resistance of *A. baumannii* to carbapenems has increasingly been reported all over the world during the last decade [2], [11], [12]. Until recently, antibiotic consumption has been pointed out as principal causative agent in acquisition of resistance genes [13]. However, this concept has been challenged since it has been discovered in 2011 a highly diverse collection of genes encoding resistance to beta-lactam, tetracycline and glycopeptide antibiotics in an authenticated ancient DNA from 30,000-year-old Beringian permafrost sediments [14]. This discovery has shown that there are reservoirs of resistance determinants that can be mobilized into the microbial community. Thus, although antibiotic resistance has long been considered as a modern phenomenon, it predates the concept of selective antibiotic pressure due to clinical antibiotic usage [14], [15].

To eventually confirm this paradigm, the objective of our study was to detect and to identify the presence of *A. baumannii* and carbapenem resistant encoding genes in natural environments in Senegal, i.e. in head lice and feces from people and pets living in different rural areas, where antibiotic pressure is believed to be low.

## Results

### Detection of *A. baumannii*

#### Head lice

From October 2010 to January 2011, 354 head lice collected from 128 women and girls (10 adults and 118 children) were analyzed and included in this study. A geographical repartition of women whose head lice were collected is presented in Figure 1. All the head lice collected were black. *A. baumannii* was detected by PCR targeting *bla*_OXA51-like_ gene in 14 head lice (4.0%) collected from 6 women (4.0%). Among these positive lice, 5 were collected in Keur Massar (12.5% of the lice collected in Keur Massar), 4 in Rufisque (7.5%), 3 in Malika (5.3%), and 2 in Dielmo (10.0%).

**Figure 1:** Head lice collection in Senegal. ***A:*** Head lice collection areas (Dakar, Kaolack, Sine-Saloum, Dielmo and Ndiop). ***B:*** Head lice collection sites in the suburbs of the Dakar region. Diamonds: number of lice positive for *A. baumannii*; green diamonds: *A. baumannii* negative for the *bla*_OXA23-like_ gene*;* red diamonds: *A. baumannii* positive for the *bla*_OXA23-like_ gene.

#### Human stool samples

The number of human stool samples tested by PCR targeting *bla*_OXA51-like_ gene for the presence of *A. baumannii* was 150 in 2008, 496 in 2009, 20 in 2010 and 51 in 2011 (Table 1). Among them, 39 were positive by PCR for *A. baumannii* (5.4%): 9 in 2008, 27 in 2009, 1 in 2010 and 2 in 2011. The majority of the positive stool samples were collected in Dielmo (29 samples). For 2011, cultivation of the 51 fresh stool specimens allowed identification of *A. baumannii* by MALDI-TOF MS in two samples, those who were positive by PCR for *A. baumannii*. Antibiotic susceptibility testing was performed, and both strains were found to be resistant to imipenem (MICs>8 confirmed using the E test). The strains were isolated from the stools of a man and a woman living in Mbao. These two isolates were also resistant to all of the other antibiotics tested, except colistin and rifampin.

**Table 1:** Repartition of stool samples and *A. baumannii*-positive stool samples.

Number of stool samples (ss) collected	Men/women/notknown	Children/adults/not known	Number of detected *A. baumannii* (locations)	bla_OXA23-like_-positive *A. baumannii*
**Year 2008 : 150 ss**				
Dielmo: 73 ss	71/79/0	150/0/0	9 (Dielmo)	0
Ndiop: 77 ss				
**Year 2009 : 496 ss**				
Dielmo: 232 ss				
Ndiop: 258 ss	222/256/18	246/222/28	27 (Dielmo: 20; Ndiop: 7)	4 (Ndiop)
Dakar: 4 ss				
Nhiakar: 2 ss				
**Year 2010 : 20 ss**				
Dielmo: 20 ss	11/9/0	11/6/3	1 (Dielmo)	0
**Year 2011 : 51 ss**				
Mbao: 28 ss				
Dominique-Pikine: 7 ss	28/23/0	22/29/0	2 (Mbao)	2 (Mbao)
Roi Baudoin: 6 ss				
IHS: 4 ss				
Saint Martin: 6 ss				

#### Animal stool samples

The presence of *A. baumannii* was searched by cultivation in stool samples from 11 donkeys, 22 cows, 9 ducks, 19 goats, 42 chickens, 8 sheep, 6 pigeons and one dog. The bacterium was isolated in seven samples (3 goats, 1 duck, 1 pigeon, 1 donkey and 1 chicken).

### Detection of the Carbapenemase-hydrolyzing Oxacillinases

All of the *bla*_OXA-51-like_-positive samples (14 head lice, 39 human and 7 animal stool samples) were checked for the presence of carbapenemase-encoding genes using PCR methods. No sample was positive for the *bla*_OXA24-like_ gene, but PCR targeting *bla*_OXA23-like_-gene was positive for 3 head lice and in 6 human stools. No animal stool sample was positive for either *bla*_OXA-like_ gene. The head lice came all from Rufisque Ouest, and the stool samples were collected in Ndiop (four samples) and Mbao (two samples). The *bla*_OXA23-like_ gene from these samples was sequenced, and the nucleotidic sequences were compared to the GenBank database using BLASTN. Of the six stool samples, all presented 100% of similarity with GenBank accession no. AJ132105. Of the three lice samples, partial nucleotidic sequences of the *bla*_OXA23-like_ gene were obtained that were 100% identical to each other and presented 100% of similarity with *bla*_OXA23-like_ sequences recently reported from groundwater samples coming from the Katmandu Valley of Nepal (GenBank accession no. AB636089). The partial translated protein sequences showed four differences in amino acid composition at positions 4, 41, 44 and 48 (Figure 2), leading to a probable new variant of *bla*_OXA23-like_ gene closely related to *bla*_OXA134_ gene from *A. radioresistens* (Figure 3). These three sequences have been deposited in Genbank under the submission ID 1538144. Unfortunately, we were not able to obtain the full sequence of this gene despite several attempts. The *bla*_OXA51-like_ gene from the two carbapanem-resistant *A. baumannii* isolated by culture in stools were also sequenced and are also presented in Figure 3. Finally, PFGE and southern blot analysis of the *bla*_OXA23-like_ gene found in the two *A. baumannii* strains isolated in the stool samples likely suggest that the gene was chromosomally encoded (Figure 4).

**Figure 2:** CLUSTAL W2 nucleotidic alignment of the three *bla*_OXA23-like_-positive *A. baumannii* found in lice (indicated louse 1 to 3) and of the six *bla*_OXA23-like_-positive *A. baumannii* found in human stool samples (indicated stool 1 to 6). The *bla*_OXA23-like_ gene AJ132105 was taken as reference.

**Figure 3:** Carbapenemase-hydrolysing oxacillinases phylogenetic tree using neighbour-joining method. *, partial *bla*OXA-23 sequences found in Uncultured *Acinetobacter* isolated from groundwater collected from deep tube well in Nepal.

**Figure 4:** PFGE and hybridization analysis. **A.** Pulsed field gel electrophoresis (PFGE) profiles obtained for the two *Acinetobacter baumannii* strains isolated from the stool samples from two patients living in Mbao. The Low Range PFG Marker (LRM) was used as molecular weight marker. **B.** Southern blot profile obtained for the two *Acinetobacter baumannii* strains isolated from the stool samples from two patients living in Mbao after hybridization against the *bla*_OXA-23 like_ DIG-labeled probe. Arrows indicate putative plasmids.

### *A. baumannii* recA Genotyping

The nine samples positive for the *bla*_OXA23-like_ gene were also sequenced for *rec*A gene. Amplifying the *rec*A gene allowed unambiguous determination of the sequence of a 336-base pair fragment. Concerning the three lice samples, all were of genotype 4 (GenBank accession no. AY274829)(11). The stool samples were all of genotype 3 (GenBank accession no. AY274828). Some samples negative for the *bla*_OXA23-like_ gene were also sequenced for the *rec*A gene and results showed that they were mostly of genotype 1 (GenBank accession no. AY274826).

## Discussion

In our work, we have shown that 4.0% of the head lice studied were positive for *A. baumannii* (14/354). The head lice being transported in alcohol, direct identification by culture could not be performed. Thus, the bacteria were detected by molecular methods only from head lice extracts with primers specific for *bla*_OXA-51-like_ gene. *A. baumannii* has previously been found in body lice collected from different European countries, from sub-Saharan African countries and from the South American continent [10], but the presence of the bacterium in lice in Senegal has not been highlighted. We have also shown that 5.4% of the human stool samples and 6.0% of the animal stool samples studied were positive for *A. baumannii*. Presence of A. baumannii in stool samples has already been shown in individuals from the community in European countries 8 but to our knowledge, environmental studies in Africa searching for the bacteria have never been performed. Our study confirmed that *A. baumannii* is not exclusively a hospital pathogen but also a nationwide human and animal colonizer.

Detection of carbapenemase encoding genes was performed on all the *bla*_OXA-51 like_ gene positive samples and results showed that 21.4% of the head lice (3/14) harbored a *bla*_OXA-23-like_ gene sequence. We believe that these sequences belong to *A. baumannii* species because, to the best of our knowledge, only *A. baumannii* species has been detected in human body lice to date. Sequencing of this gene allowed discovering a putative new variant but unfortunately we were unable to obtain the full sequence of this gene. Interestingly, our sequence was 100% identical to *bla*_OXA23-like_ partial sequences found recently by Tanaka *et al*. in groundwater samples coming from the Katmandu Valley of Nepal, showing presence of multi-drug resistant *Acinetobacter* in different environments in the world [16]. These sequences are closely related to *bla*_OXA134_ gene from *A. radioresistens* (Figure 3). Carbapenem-resistance encoding gene sequences have never been detected previously in human lice. Until now, the *A. baumannii* isolates detected in human lice were remarkably susceptible to antibiotics, particularly to carbapenems [10], as shown by the sequenced SDF strain isolated from a human body louse. Analysis of its genome showed a remarkably susceptible strain that harbored several hundred of Insertion Sequence elements [17] that might play a role in the acquisition of carbapenem-resistant genes in *A. baumannii*. Thus, it would be necessary, in future studies, to cultivate the samples in order to isolate the bacteria and to fully characterize this carbapenemase encoding gene.

Besides, our study was the first to show the presence of carbapenem-resistant *A. baumannii* isolates in human stool samples in Senegal. Carbapenem resistance, which has been detected by antimicrobial susceptibility testing, was associated with resistance to all of the beta-lactams and to most of the antibiotics tested. Resistance to carbapenems has been characterized at the molecular level with specific primers targeting two oxacillinase genes and here, *bla*_OXA-23-like_ was detected. Multidrug-resistant (MDR) *A. baumannii* strains producing oxacillinase enzymes have been reported worldwide, especially in nosocomial outbreaks [1], [2], [18], [19]. These facts have been evidenced by the large number of studies published [1], [2], [20]. However, concerning the epidemiology of MDR *A. baumannii* in African countries, only a few studies have been performed. MDR strains have been isolated in Tunisia [21], Algeria 19,22,23, Namibia and South Africa [24]. What was intriguing in our study was that carbapenemase encoding genes were detected in environmental samples where antibiotic pressure was low. Some explanation might be brought by D’Costa *et al*., who recently discovered reservoirs of resistance determinants in environments like permafrost sediments that were free from antibiotic contamination [14], showing that antibiotic resistance predates the concept of selective antibiotic pressure due to clinical antibiotic usage. It has also been shown that soil-dwelling bacteria produced and encountered a myriad of antibiotics, and that they are a reservoir of resistance determinants that can be mobilized into the microbial community 25. Although there was no doubt that bla_OXA23_ gene was present in *A. baumannii* species for the two human stool isolates in our study, we could not exclude the possibility that samples only analyzed by PCR methods that were positive for bla_OXA51_ and bla_OXA23_ could be due to the combination of *A. baumannii* with another *Acinetobacter* spp. harboring bla_OXA23._ Although *bla*_OXA-23-like_ gene was likely transferred in environment from a reservoir that is unknown here, gene transfer from the environmental bacterium *Acinetobacter radioresistens* has been previously described by Poirel *et al*. [26]. More recently, the presence of the bla_OXA23-like_ gene has also been detected in *Acinetobacter* genomospecies 15TU isolates found in rectal samples collected from cattles in France, suggesting potential gene exchanges [27]. Our suppositions are supported by the fact that lateral gene-transfer are common and can be important mechanisms in genome evolution [28]. Moreover, one can question on the presence of genetic mobile elements in *A. baumannii*, that have shown to play a key role in regulatory changes [29].

Finally, the *rec*A genotypes of the *A. baumannii* found in the bla_OXA23-like_ –containing samples were limited to two clones. One clone was detected only in lice that were collected in Rufisque (east of Dakar), and the other one was detected only in stools that were collected in Ndiop (South of Dakar) and Mbao (east of Dakar, near Rufisque). Thus, *A. baumannii* genotypes were specific to the sample origin and not distributed geographically.

In summary, our study showed the presence of a reservoir of *A. baumannii* carbapenem-resistant isolates in human stools collected in Senegal, in places where it is unlikely that they have been selected by antibiotic prescriptions. Finally, our results question the breadth of *A. baumannii* reservoirs and the cause of the carbapenem resistance beyond antibiotic pressure.

## Materials and Methods

A part of this study concerns the Dielmo project, a longitudinal prospective study initiated in 1990 for long-term investigation of host-parasite relationships [30], [31].

### Sample Collection

Head lice were collected from October 2010 to January 2011, from women with no clinical symptoms from different locations in Senegal (Figure 1). Lice collected in Ndiop were preserved in alcohol; the others were kept in dry tubes. All of them were transferred to Marseille (France) at room temperature. The human stool samples included in this study were collected from 2008 to 2010 in Dielmo and Ndiop, Senegal, from healthy persons, as previously described [32], and mixed with 2.5 mL of absolute ethanol for storage and transportation to Marseille at room temperature. In 2011, 51 diarrheal stool samples were also collected in Dakar (Senegal) and cultivated on Drigalski and sheep blood agar media. In addition, free stool samples were collected immediately after defecation to decrease the risk of contamination from soil by local farmers on their own domestic and wild animals in the area of Dielmo and Ndiop and cultivated. No experimentation was done on these animals. Bacterial identification at the species level was performed on each colony obtained on the culture media using the Matrix-assisted Laser Desorption Time-of-Flight Mass Spectrometry (MALDI-TOF MS) (Microflex, Bruker Daltonics) with the flex control software (Bruker Daltonics). A score value >1.9 was considered positive for identification at the species level, as previously reported [33].

### Susceptibility Testing

For the *A. baumannii* strains isolated in human and animal stool samples in 2011, antibiotic susceptibility testing was performed by the disc diffusion method using a panel of 14 different antibiotics including ticarcillin-clavulanic acid, piperacillin-tazobactam, ceftazidime, imipenem, ciprofloxacin, amikacin, gentamicin, tobramycin, sulfamethoxazole-trimethoprim, colistin and rifampicin [18]. Susceptibility breakpoints used were those recommended by EUCAST (www.eucast.org). According to EUCAST breakpoints, an isolate is considered resistant or susceptible to imipenem with inhibition diameters <17 mm and ≥23 mm, respectively. For isolates with diameters <17 mm, Minimum Inhibitory Concentrations (MICs) were determined using the E test method (AB Biodisk, Solna, Sweden), and resistance was defined as isolates with MIC against imipenem >8 mg/L.

### Molecular Detection of Carbapenemase-hydrolyzing Oxacillinases

Genomic DNA was extracted from bacterial colonies identified as *A. baumannii* by MALDI-TOF MS, as described above. Concerning the lice, each was previously rinsed twice in sterile water for 15 minutes. Total genomic DNA from each half louse and all stool samples collected was extracted using the BioRobot MDx workstation (QIAGEN, Hilden, Germany) in accordance with the manufacturer’s recommendations and protocols. The detection of *A. baumannii* was determined by screening the samples (lice and stool) with a real-time PCR assay targeting the *bla*_OXA51-like_ gene (Table 2). Amplification was performed using thermocycler conditions as follows: an initial denaturation step at 95°C for 15 min followed by 40 cycles of denaturation at 95°C for 30 sec and extension at 60°C for 1 min. Negative and positive controls were included in each assay. For all the samples positive for *bla*_OXA51-like_ gene, molecular detection and sequencing of the carbapenemase-encoding genes *bla*_OXA23-like_ and *bla*_OXA24-like_, the two most common carbapenemase-encoding genes in *A. baumannii*, was performed by PCR. The presence of *bla*_OXA58_ gene was not investigated in this study. The conditions used for detection are as follows: an initial denaturation step at 95°C for 15 min followed by 40 cycles of denaturation at 95°C for 30 sec, hybridization at 57°C for 30 sec and extension at 72°C for 1 min, and a final extension at 72°C for 10 min. (Table 2). Finally, the *bla*_OXA51-like_ gene was sequenced for carbapenem-resistant *A. baumannii* isolated by cultivation.

**Table 2:** Oligonucleotide primers and TaqMan* fluorescent probe sequence used for PCR and sequencing of *Acinetobacter baumannii.*

Targets	Primer Names	Primer Sequences	Amplicon Size (bp)	References or sources
	OXA51_like_-F	5′-AACATTAAAGCACTCTTACTTATAAC		This study
bla_OXA51-like_	OXA51_like_-R	5′-TTGTTGGATAACTAAAACACCCGT	171	
	OXA51_like_-Dye	FAM-TGCTCACCTTATATAGTGTCTGCTAA-TAMRA		
	OXA51_like_-FSeq	5'-TAATGCTTTGATCGGCCTTG	353	
bla_OXA51-like_	OXA51_like_-RSeq	5'-TGGATTGCACTTCATCTTGG		[34]
bla_OXA23-like_	OXA23_like_-F	5′-GATCGGATTGGAGAACCAGA	501	[35]
	OXA23_like_-R	5′-ATTTCTGACCGCATTTCCAT		
bla_OXA24-like_	OXA24-F	5′-ATGAAAAAATTTATACTTCCTATATTCAGC	825	[36]
	OXA24-R	5′-TTAAATGATTCCAAGATTTTCTAGC		
*rec*A	rA1F	5′-CCTGAATCTTCTGGTAAAAC	424	[10]
	rA2R	5′-GTTTCTGGGCTGCCAAACATTAC		

* Applied Biosystems, Courtaboeuf, France.

### *A. baumannii* recA Genotyping

For samples positive for carbapenemase-hydrolyzing oxacillinases, the *rec*A gene was amplified and sequenced using specific primers as previously described [10] (Table 2). Some negative samples were also selected for *rec*A genotype determination. Genotypes were determined by comparing *recA* sequences with the genotypes deposited in the GenBank database.

### Carbapenemase-encoding Genes Analysis by PFGE and Hybridization

*A. baumannii* genomic DNA plugs were performed and equilibrated in 0.5×TBE (50 mM Tris, 50 mM boric acid, 1 mM EDTA). Each agarose block as well as molecular weight markers (Low Range PFG Marker and Lambda Ladder PFG Marker – Biolabs, New England) were placed in the well of a 1% PFGE agarose gel (Sigma). The pulsed field gel separation was made on a CHEF –DR II apparatus (Bio-Rad Laboratories, Inc) with pulses ranging from 2 to 20 seconds at a voltage of 5 V/cm and switch angle of 120° for 22 hours at 14°C. Gels were stained with ethidium bromide and analyzed using a Gel-Doc 2000 system (Bio-Rad Laboratories) and used to prepare Southern blots. The gel was transferred onto Hybond N+ (GE Helathcare) with the vacuum blotter (model 785, Bio-Rad) and UV cross-linked for 2 min. The blots were then hybridized against the Oxa-23 DIG-labeled probe (Table 2) as recommended by the manufacturer (DIG-System, Roche Diagnostics) except that detection of the hybridized probe was performed using a horseradish peroxidase-conjugated monoclonal Mouse Anti-Digoxin (Jackson Immunoresearch, 1∶20 000). After washings, blots were revealed by chemiluminescence assays (ECL, GE Healthcare). The resulting signal was detected on Hyperfilm™ ECL (GE Healthcare) by using an automated film processor (Hyperprocessor™, GE Healthcare).

### Ethic Statement

Informed verbal consents were obtained from all the participants involved in our study. This study was approved (Agreement #11-010), by the Ethic Committee of the Institute Fédératif de Recherche 48, Marseilles, France since this study was a non-interventional epidemiological research study as a part of the French Bioethics law N° 2004-800 (06/08/2004). In addition, free stool samples were collected from soil by local farmers on their own domestic and wild animals in the area of Dielmo and Ndiop and cultivated and no experimentation was done on these animals.
